The article "Intra‐day variations in volar forearm skin hydration" was published in 2024. Journal: Skin Res Technol.

# Intra‐day variations in volar forearm skin hydration

**DOI:** 10.1111/srt.13849

**Published:** 2024-07-08

**Authors:** Harvey N. Mayrovitz

**Affiliations:** ^1^ Department of Medical Education, Dr. Kiran C. Patel College of Allopathic Medicine Nova Southeastern University Fort Lauderdale USA

**Keywords:** arm skin, gender differences, skin hydration, skin temperature, skin water, tissue dielectric constant, whole body fat, whole body water, young adults

## Abstract

**Background:**

Skin hydration (SKH) measurements are used for multiple purposes: to study skin physiology, to clinically investigate dermatological issues, and to assess localized skin water in pathologies like diabetes and lymphedema. Often the volar forearm is measured at various times of day (TOD). This report aims to characterize intra‐day variations in volar forearm SKH to provide guidance on expected TOD dependence.

**Materials and methods:**

Forty medical students (20 male) self‐measured tissue dielectric constant (TDC) on their non‐dominant forearm in triplicate as an index of local skin tissue water every 2 h starting at 0800 and ending at 2400 h. All were trained and pre‐certified in the procedure and had whole‐body fat (FAT%) and water (H_2_O%) measured. Day average TDC (TDC_AVG_) was determined as the average of all time points expressed as mean ± SD.

**Results:**

Males versus females had similar ages (25.1 ± 2.2 years vs. 25.1 ± 1.5 years), higher H_2_O% (56.6 ± 5.0 vs. 51.8 ± 5.7, *p* = 0.002), and higher TDC_AVG_ (32.7 ± 4.1 vs. 28.5 ± 5.1, *p* = 0.008). TDC values were not significantly impacted by H_2_O% or FAT%. Female TDC exhibited a significant decreasing trend from morning to night (*p* = 0.004); male TDC showed no trend.

**Conclusion:**

Skin water assessed by TDC shows some intra‐day variations for females and males but with quite different temporal patterns. Clinical relevance relates to the confidence level associated with skin hydration estimates when measured at different times of day during normal clinic hours which, based on the present data, is expected to be around 5% for both males and females.

## 1 INTRODUCTION

Skin hydration measurements are used in skin research to uncover basic features of skin physiology,^1^to clinically assess features of relevant dermatological issues such as atopic dermatitis,^2^, ^3^, ^4^ psoriasis,^5^, ^6^ ichthyosis^7^ and wound healing^8^, ^9^, ^10^ and also to assess localized skin water relevant to other pathologies including those present in diabetes mellitus^11^, ^12^, ^13^ and breast cancer related lymphedema.^14^, ^15^, ^16^ Often the volar forearm is the target of such measurements.^17^, ^18^, ^19^ Because these measurements can often be made at different times during the day, it would be useful to have an estimate of how much variability to expect when skin hydration values are obtained at differing times. It would also be of interest to determine the possible role of gender and body habitus parameters in this process. Some initial pioneering inroads have been made in the assessment of the temporal variability^20^, ^21^, ^22^ as has been recently reviewed.^23^, ^24^ The present report focuses more deeply on this issue by assessing local skin hydration via tissue dielectric constant (TDC) measurements obtained every 2 h from 0800 to 2400 h in 40 healthy young adults equally divided by gender.

The article "Intra‐day variations in volar forearm skin hydration" was published in 2024. Journal: Skin Res Technol.

## 2 METHODS

### 2.1 Subjects

Forty young healthy adult medical students, equally divided by gender, participated in this self‐measurement research that was approved by the Nova Southeastern University Institutional Review Board. To be part of the study, subjects needed to agree to be successfully trained in needed measurement methods and to be willing and able to do self‐measurements at 2‐h intervals from 0800 to 2400 h on a single day of their choice. Exclusions to participation were any skin conditions or open wounds affecting forearm skin.

### 2.2 Measurements

TDC was measured to an effective depth of between 2.0 and 2.5 mm using the MoistureMeterD Compact (Delfin Technologies, Kuopio Finland). This device operates at a frequency of 300 MHz and functions as an open‐ended coaxial transmission line,^25^, ^26^, ^27^, ^28^ to determine TDC that largely depends on water content within the measurement volume.^29^, ^30^ The method has been validated,^31^ and shown to be reliable.^32^, ^33^, ^34^ Measurements are done by touching the skin with the device for a few seconds as illustrated in Figure 1. Whole body fat and water percentages (FAT% and H_2_O% respectively) were measured using bioimpedance at 50 KHz (InnerScan Body Composition Monitor, Tanita model BC558, The Competitive Edge, Vancouver, WA, USA). Body composition measurements were made after the subject removed their footwear and stood on a scale for about 10 s while gripping a handle‐electrode as illustrated in Figure 2. Weight, FAT% and H_2_O% were measured as previously described that is determined by a device priority algorithm.^35^ Skin temperature (TSK) at the site of TDC measurements was measured using an infrared non‐contact device (Exergen, Watertown Main, USA, Model DX501‐RS) with a stated repeatability of ± 0.1°C. Room temperature (TRM) and relative humidity (RH) were also measured (Fluke Model 971, Everett, WA, USA, with a stated accuracy of ± 0.1°C for TRM and ± 2.5% for RH.

**FIGURE 1:** Self‐measurement of TDC. TDC is measured on the forearm of the non‐dominant hand in triplicate at a site located five cm distal to the antecubital fossa. As shown, the digital display indicates the PCW. For the data presented in the text the actually measured TDC value is used. These are related via the approximate equation TDC = 0.8 × PCW. PCW, percentage water; TDC, tissue dielectric constant.

The article "Intra‐day variations in volar forearm skin hydration" was published in 2024. Journal: Skin Res Technol.

**FIGURE 2:** Measuring whole body fat and water percentages. Body composition measurements (Weight, whole body fat percentage, and whole body water percentage) were made after the subject removed their footwear and stood on the impedance scale for about 10 s while gripping a handle‐electrode as illustrated.

### 2.3 Initial procedures

Prior to starting self‐measurements each potential participant was trained and evaluated in the proper use of each skin measuring device by the author during a dedicated training session. During that session, but following their individual training, each participant performed a series of measurements that replicated what they would do during their self‐measurement protocol. This sequence of measurements was observed for proper technique and if needed corrected and a second sequence was carried out. No participant required any further corrections. At the conclusion of this training and validation session the total body weight, FAT%, and H_2_O% were measured as described in the methods section.

### 2.4 Self‐measuring procedure

The self‐measurer performed their measurements on the day when they were to be at home for the entire day. This was almost always a weekend day. All measurements were done on the nondominant forearm while they were seated with the forearm supported on a suitable table surface. During the measurement day, no lotions, creams, or other substances were permitted to be applied to the forearm skin. The measurement site, which was on the volar forearm five cm distal to the antecubital fossa, was marked with a small dot using a surgical pen. TDC was measured in triplicate at this site followed by a measurement of TSK at the same site. Then TRM and RH were recorded. This sequence was repeated every 2 h starting at 0800 h and continuing to and including 2400 h constituting nine sequential measurement cycles over 16 h. During the entire sequence, the measurer's activities were confined to normal ones that consisted mostly of studying, watching TV, listening to music, and at times eating and drinking non‐caffeinated beverages. No vigorous activity was permitted nor was washing of the forearm permitted.

### 2.5 Analysis

The triplicate TDC values were averaged to yield one TDC value for each measurement event for each subject, resulting in 40 TDC values per measurement time. These values were tested for normality via the Shapiro–Wilk test at each measurement time. These tests indicated that normality could not be assumed for at least two of nine intervals. Tests for normality of the male and female groups separately showed that for six measurement times normality could not be assumed. Thus, to test for potential differences in TDC values among the nine measurement times, the nonparametric Friedman test was used. When comparing male versus female parameters the nonparametric Mann‐Whitney test was used. All statistical tests were done using SPSS, version 16. To evaluate if body habitus parameters (BMI, FAT%, and H_2_O%) impacted TDC values, the per person time average TDC value (TDC_AVG_) was determined as the average TDC value over all nine measured times. TDC_AVG_ was then compared between subgroups who had body habitus parameters below and above their median values. Comparisons between these two subgroups were based on the Mann–Whitney test.

The article "Intra‐day variations in volar forearm skin hydration" was published in 2024. Journal: Skin Res Technol.

## 3 RESULTS

### 3.1 Subject characteristics

Table 1 summarizes the main demographic features of the male and female participants. Male and female participants had similar ages that ranged from 22 to 30 years with a mean ± SD of 25.1 ± 1.8 years for the entire group (*N* = 40). Males compared to females had a greater BMI (*p* = 0.001), greater total body water percentage (*p* = 0.002), and less fat percentage (*p* = 0.038). It was notable that 50% of the males were either overweight or obese compared to only 10% females. Except for two participants (one male and one female), the non‐dominant hand was the left hand.

**TABLE 1:** Demographic comparisons by gender.

	Female	Male	*p*‐value
*N*	20	20	
Age (years)	25.1 ± 2.2	25.1 ± 1.5	0.883
Height (cm)	162.9 ± 7.9	180.0 ± 5.5	< 0.001
Weight (Kg)	60.4 ± 13.5	86.5 ± 16.8	< 0.001
BMI (Kg/m^2^)	22.7 ± 4.8	26.0 ± 5.4	0.001
Fat%	31.1 ± 7.8	24.2 ± 9.5	0.038
H_2_O%	51.8 ± 5.7	56.6 ± 5.0	0.002

BMI Classification			
%Underweight (BMI < 18.5 Kg/m^2^)	0	5	
%Normal weight (BMI 18.5−24.9 Kg/m^2^)	90	45	
%Overweight (BMI 25.0–30.0 Kg/m^2^)	5	35	
%Obese (BMI > 30 Kg/m^2^)	5	15	

Race/Ethnicity			
% White/Caucasian	40	55	
%Asian‐Indian	20	15	
%Asian‐East	20	5	
%Hispanic	15	20	
%Middle East	5	5	

*Note*: Variable entries are the mean ± SD or percentages. *p*‐Values are based on the nonparametric Mann–Whitney test. Note that 50% of the males were either overweight or obese compared to only 10% of females. Fat% was greater and water% less in females. Race/Ethnicity was based on the self‐report of participants.

### 3.2 Temperature and humidity variation among time‐of‐day

Figure 3 shows the pattern of variation among time‐of‐day as measured at 2‐h increments. Tests for significant differences among times using the nonparametric Friedman test failed to detect a significant difference in room temperature, skin temperature, or room relative humidity over the 16‐h measurement interval. Averaging of these values over the nine measurement times yielded an overall average ± SD for TRM_AVG_, TSK_AVG_, and RH_AVG_ of 20.9 ± 2.3°C, 32.1 ± 1.2°C, and 54.8 ± 8.3%, respectively. TSK_AVG_ did not significantly differ between males and females (*p* = 0.871).

The article "Intra‐day variations in volar forearm skin hydration" was published in 2024. Journal: Skin Res Technol.

**FIGURE 3:** Temperature and humidity conditions. Data points are the mean and SD for room RH, TRM, and TSK at the forearm measurement site. Dashed lines indicate the linear regression trend of the group mean values (*N* = 40). No significant difference in any parameter among times was detected as determined based on the Friedman test. RH, relative humidity; SD, standard deviation, TRM, room temperature; TSK, skin temperature.

### 3.3 TDC variation among time‐of‐day

For males the difference between TDC values among time was not statistically significant (*p* = 0.091) whereas for females there was a decrease in TDC as the day progressed (*p* = 0.004). The pattern of TDC versus time of day is shown in Figure 4. The figure displays the group mean TDC values versus time along with the standard error of the mean (SEM).

**FIGURE 4:** TDC versus time of day. Data points are the mean value of each group and error bars are the SEM. TDC variation among times for females is statistically significant based on the Friedman test (*p* = 0.004) but males are not (*p* = 0.091). Dashed lines indicate the linear regression trend of the group mean values. At every time point the male TDC values were greater than the female values with the *p*‐values at each time indicated in the graphic. SEM, standard error of the mean; TDC, tissue dielectric constant.

Considering all measured TDC values the overall TDC_AVG_ was greater for males than females (32.7 ± 4.1 vs. 28.5 ± 5.1, *p* = 0.008). This difference represents a 14.7% lower TDC_AVG_ for females. Although female TDC values decrease linearly with time, the magnitude of the decrease from 0800 to 2400 h was 6.5%. The decrease from 0800 to the usual end of clinic measurement days (1800 h) was 4.7%. Alternatively, if the maximum difference between any two time points for each subject is determined, the female group average difference was 3.4 ± 2.8. For males, although there was no significant trend or overall difference in TDC values among times, there were still differences in TDC values as measured at different times. The maximum difference in mean TDC values was between 1400  and 1800 h which amounted to 4%. Alternatively, if the maximum difference between any two time points for each subject is determined, the male group average difference was 3.8 ± 2.8. There was no consistent time at which the maximum or the minimum values occurred for male TDC values.

The article "Intra‐day variations in volar forearm skin hydration" was published in 2024. Journal: Skin Res Technol.

### 3.4 TDC dependence on body habitus parameters

Comparison of TDC_AVG_ between subgroups who had BMI, FAT%, and H_2_O% values below or above the median values did not reveal any statistically significant differences in TDC_AVG_ between males or females for any parameter as summarized in Table 2. For both sexes, there was a tendency for subjects with higher FAT% to have lower TDC values and for subjects who had higher H_2_O% to have higher TDC values.

**TABLE 2:** TDC values by body habitus parameters.

	Females				Males			
	Parameter Median Value	TDC_AVG_ below median	TDC_AVG_ above median	*p*‐value	Parameter Median Value	TDC_AVG_ below median	TDC_AVG_ above median	*p*‐value
BMI (Kg/m^2^)	21.95	28.0 ± 5.3	29.0 ± 5.0	0.853	25.15	34.2 ± 4.9	31.1 ± 2.4	0.123
Fat%	29.8	29.8 ± 7.3	27.4 ± 1.9	0.604	20.4	34.0 ± 4.7	31.4 ± 3.2	0.247
H_2_O%	52.4	28.0 ± 2.8	29.0 ± 6.8	0.968	56.8	31.5 ± 3.2	33.8 ± 4.7	0.315

*Note*: Table entries show the median value for each body habitus parameter (BMI, FAT%, and H_2_O) and the TDC_AVG_ for subject subgroups who had parameters below and above these median values. TDC_AVG_ is shown as mean ± SD. *p*‐Values are based on the nonparametric Mann‐Whitney test. FAT% and H_2_O% are whole body fat and water percentages.

Abbreviations: TDC_AVG_, average TDC value; TDC, tissue dielectric constant.

## 4 DISCUSSION

Evidence consistent with a reduction in skin water from morning to afternoon was reported based on skin ultrasound measurement changes in skin thickness.^36^ In that study of young adult healthy men and women, skin thickness was measured two times, one in the morning between 0830–1030 and then again between 1530–1700. Forearm skin thickness was reported to decrease in both males (*N* = 20) and females (*N* = 20) and this change was attributed to a diurnal redistribution of water. Skin thickness measurements were also done on face areas with a similar finding and on lower extremities with opposite findings. Other work on a group of 23 elderly (ages 75–100) nursing home residents also reported a diurnal change in forearm skin thickness that might be attributed to redistribution of fluid from morning to evening in the aged skin.^37^ One study used ultrasound low echogenicity patterns as an index of skin water and also reported patterns consistent with diurnal changes in 22 young adults (16 female) but not in 22 elderly persons (16 female).^22^ In these studies, skin water content was not actually measured. However, in a small study of 12 females in whom skin water was self‐measured based on skin TDC values every hour between 0800 and 2000, similar findings were reported in which both facial and forearm skin water decreased from morning to evening whereas lower extremity skin water increased.^38^ The present results extend these prior findings with respect to intra‐day forearm skin water changes based on direct TDC measurements and by considering both females and males in equal numbers as well as considering the potential impact factors of skin temperature and body habitus evaluated at multiple times during the day.

The article "Intra‐day variations in volar forearm skin hydration" was published in 2024. Journal: Skin Res Technol.

The main findings of the present study indicate no significant time dependent intra‐day trend in forearm TDC values for males although when considering the group mean maximum at 1400 h and the group mean minimum at 1800 h a TDC difference of 4% was determined. Contrastingly, for females, a statistically significant decline in TDC values was observed from 0800 to 2400 h with a mean decrease of 6.5% between these time points. These patterns were not significantly impacted by skin temperature or body habitus parameters that included body mass index and total body fat and water percentages. As has been reported in other contexts,^35^ the present result also confirmed the greater TDC values of male versus female skin, in the young adult population herein evaluated. Potential causes of this difference are beyond the present scope of investigation but have been previously discussed in which the possibility of its relationship to the greater male dermis thickness and lesser low water content fat of the forearm largely explain the greater TDC values.^39^, ^40^

However, what remains unexplained based on the present findings is the gender difference in the intra‐day TDC variation. The decrease in TDC from morning through evening, herein observed in the female group, may be explained on the basis of a gravitationally related shift in overall water distribution that impacts skin water. This concept has been put forward by others and may play a role especially as it relates to the lower part of the body.^36^ However, one would expect such forces to be present in both genders, but at least in the present study, this is not what was observed in the forearms.

In a search for alternate explanations, one may look at the possibility of gender‐related differences in transepidermal water loss (TEWL). In a study that assessed TEWL in a small group of eight males and nine females, TEWL of forearm skin was reported to decrease by 7.2% over an 8 h period with the male rate being 5% greater than for females.^41^ Such a decrease in TEWL would not be expected to be associated with a decline in TDC over the same interval, so that temporal changes in TEWL may not explain the present findings.

The article "Intra‐day variations in volar forearm skin hydration" was published in 2024. Journal: Skin Res Technol.

However, differences in male versus female absolute TEWL rates might be involved, but the literature on this point is conflicting. In a large group of 150 males and 150 females, a significantly lower TEWL was observed in males compared with females up to the age of about 50 years.^1^ The higher TEWL in the females might partially explain the observed decline in TDC over the 16‐h interval. However, arguing against this possible explanation are reports of TEWL being greater in males compared to females in the forearm^17^ and the face.^42^ Hence the explanation of the differential pattern of TDC variation with time‐of‐day herein observed between males and females must await clarification via other research studies.

Although the decline in TDC through the day in females is unexplained, from a clinical perspective, the present findings document the amount of variation to be expected in both genders, which should help in estimating the potential importance of small differences if measured at a different time of the day.

### 4.1 Study limitations

One limitation of the present study is the fact that the data obtained is based on self‐measurements done by multiple persons. Although each participant was trained and certified in the measurement and protocol process by the author, this does not guarantee that, when not observed, errors may occur. However, the consistency of the data among all participants, which was carefully reviewed, suggests that any deviations would have been small and limited in overall effect considering the reasonable number of individual participants.

The present findings apply specifically to the young adult healthy population herein studied and potential generalizations to either older populations or persons with conditions such as arm edema or lymphedema would require further verification. However, the results call attention to the possible gender differentials that should be taken notice of and also to the consideration of time‐of‐day for evaluation that applies to all persons being tested.

## 5 CONCLUSION

Skin tissue water assessed by TDC values shows minor intra‐day variations for both females and males. However, the pattern of changes between genders is different with a significant decreasing trend from morning to evening in females but not in males. The explanation for this difference is not provided by the present data but it is suggested that gender differences in TEWL may be involved. TDC values for both genders were not dependent on whole body water or fat percentages, but at all times of day male TDC values significantly exceed female values. In part the clinical relevance of the findings relates to the confidence level associated with skin hydration estimates when measured at different times of day during normal clinic hours, which based on the present data is expected to be around 5%.

The article "Intra‐day variations in volar forearm skin hydration" was published in 2024. Journal: Skin Res Technol.

## Data Availability

The data that support the findings of this study are available on request from the corresponding author. The data are not publicly available due to privacy or ethical restrictions.
